The article "Design of Cloud Storage-Oriented Sports Physical Fitness Monitoring System" was published in 2022. Journal: Comput Intell Neurosci.

# Design of Cloud Storage-Oriented Sports Physical Fitness Monitoring System

**DOI:** 10.1155/2022/1889381

**Published:** 2022-06-10

**Authors:** Zhou Zheng, Yang Liu

**Affiliations:** ^1^Hulunbuir University, Institute of Physical Education, Inner Mongolia, Hulunbuir 021008, China; ^2^Physical Education Institute of Shanxi Normal University, Shanxi 710119, China

## Abstract

In order to improve the accuracy and response speed of sports fitness monitoring results and make the monitoring results more comprehensive, a new cloud storage-oriented sports fitness monitoring system is designed. Based on cloud storage technology, the overall framework of the sports fitness monitoring system is established; the function of the hardware module of the monitoring system is analyzed, and distributed database is established. The ray-casting image feature scanning method was used to collect the physical condition monitoring image and generate a high-quality human body target frame to realize the physical condition monitoring. Based on the monitoring data, the fitness method recommendation method is designed according to the user's physical condition. The experimental results show that the monitoring results of the proposed system have higher accuracy, faster system response speed, and higher comprehensiveness of the monitoring results, which verifies the application value of the proposed system.

## 1. Introduction

With the application of computer-related technology in the field of sports [1], sports-related units at all levels have established their own sports information management or sports physical fitness monitoring management systems to systematically manage relevant data [2, 3]. However, at present, the physique data databases established by various units are isolated from each other. Moreover, due to the mobility of the population, it brings great inconvenience to large-scale and effective physique monitoring, longitudinal tracking research, and personal understanding of their own physique [4, 5]. At the same time, how to use the data of national physique monitoring to scientifically guide the national fitness and apply the national physique monitoring results to practice is also the focus and development direction of physique monitoring research [6]. In order to more conveniently manage and utilize the research results in the field of sports science such as national physique monitoring, promote the transformation of the research results of physique monitoring into practical application results, and facilitate individuals to get the feedback and scientific guidance of physique test results in time, it is urgent to establish a sports physical fitness monitoring system [7, 8].

Reference [9] designs an autonomous fitness monitoring system based on a monocular camera, which relies on the monocular camera of a mobile phone and 3D human key point detection technology to monitor whether the fitness actions of users are standard in real time and give corresponding prompts through voice. The monitoring effect of the system is verified by comparing with the related work in recent years. The results show that the system can accurately evaluate fitness movements in real-time monitoring, but there is a problem of long system response time. Reference [10] designed a video monitoring system for children's sports training based on feature moving frame differential scanning and adaptive compensation. The Internet of Things networking technology was used to collect video monitoring images of children's sports training, and the three-dimensional data field of three-dimensional reconstruction of video monitoring images of children's sports training was constructed. According to the distribution characteristics of the data field, the physical condition of sports training can be monitored to analyze the video monitoring images of children's sports training and extract the physical condition characteristics. The experimental results show that the real-time performance of the system is poor, and the accuracy of the monitoring results is low. Reference [11] based on Taubin smoothing filter designed a children's sports training image 3D reconstruction of video monitoring systems and children's sports training video monitoring of the surface of the image of 3D reconstruction, according to the result of the reconstruction of physical conditions of sports training in real-time monitoring, but this method is not suitable for monitoring image interference intensity bigger. The response speed cannot meet the real-time requirements, and the monitoring results are not comprehensive enough.

To solve the above problems, this paper designs a sports physical fitness monitoring system for cloud storage. The main research contents are as follows:

1. Under the support of cloud storage technology, establish the sports physical fitness monitoring system, establish the system application support platform by using a series of network interconnection and information security technologies, and ensure the safe and reliable transmission of sports physical fitness monitoring information by using firewall technology and data encryption technology.
2. The hardware module of the monitoring system is divided into five functional modules: knowledge base management module, perception module, physical fitness data sampling module, physical fitness project information management module, and parameter setting module, and the function of each module is analyzed.
3. The ray casting image feature scanning method is used to collect the monitoring image of physical condition in sports training. The image convolution, clipping, translation, scaling, and rotation are given through the spatial transformation network, so that the moving target has spatial invariance, and the image data can be automatically transformed in space to generate a high-quality human target frame to realize the monitoring of the physical condition.
4. After realizing the sports physical fitness monitoring, take the monitoring data as the basis, design the fitness mode recommendation method according to the user's physical fitness state, and improve the practical application value of the system.
5. Finally, simulation experiments are carried out to show the advantages of the proposed system in improving the sports physical fitness monitoring ability.

## 2. Design of Sports Physical Fitness Monitoring System

### 2.1. Overall Structure and Supporting Platform Design of Sports Fitness Monitoring System

#### 2.1.1. Overall Structure of Sports Physical Fitness Monitoring System

Cloud storage technology [12, 13] is a networked storage concept rising in recent years. It is an emerging technology derived and developed on the basis of cloud computing [14, 15]. Cloud storage is a mode of online storage, that is, data are stored on multiple virtual servers usually hosted by a third party, rather than exclusive servers. Hosting companies operate large data centers. People who need a data storage and hosting can meet the needs of data storage by purchasing or renting storage space from them. According to the needs of customers, data center operators prepare storage virtualized resources at the back end and provide them in the form of a storage resource pool, so that customers can use this storage resource pool to store files or objects by themselves. In fact, these resources may be distributed on many server hosts, which is also the theoretical basis of cloud storage analysis. Combined with developed Internet technology, advanced cluster application, and mature distributed file system, this technology enables the massive types of storage devices in the network to work together to form an overall storage and computing structure model and jointly provide data storage and computing services and interface access functions. This paper transmits the collected data to the cloud platform through the wireless network to realize the cloud storage function [16], which can realize the storage and calculation of massive sports fitness monitoring data. In addition, compared with embedding the algorithm into the sensor terminal module program, the data processing algorithm stored on the remote cloud platform can be continuously optimized and updated in real time to ensure the accuracy and expansibility of the data [17, 18].

According to the characteristics of sports fitness monitoring, relying on cloud storage as the bottom end, through B/S and C/S multilayer architecture, realize the overall architecture design of the sports fitness monitoring system. The overall architecture of the system is shown in Figure 1.

According to Figure 1, based on the architecture of “optical fiber sensing terminal + data processing relay + cloud platform + heterogeneous application terminal” [19, 20], combined with cloud storage technology, the sports fitness monitoring system designs a system framework including sensing layer, cloud platform, management layer, data processing layer, and application layer.

#### 2.1.2. System Application Support Platform

The network application support platform uses the TCP/IP protocol as the network communication protocol and is composed of network servers, communication equipment, security equipment, etc., and applies the latest, the most advanced network core technology also includes existing network application support systems and supports the operation of the upper-layer application software. Establish a safe, stable, reliable, and open network application platform, which is the cornerstone of establishing a comprehensive management environment for sports physical fitness monitoring information.

The network application support platform, based on open protocols and technical standards, is not limited to any hardware platform or network platform, spanning Unix, Windows NT, and other network operating systems and realizing multiplatform, multiprotocol, and multioperating system communication. This feature makes the comprehensive environment for sports physical fitness monitoring information management independent of the network environment, and the network application support platform is completely transparent to the application system to ensure a seamless connection between different systems.

The network application support platform adopts a series of network interconnection and information security technologies, uses firewall technology and data encryption technology to ensure the safe and reliable transmission of sports physical fitness monitoring information, and more importantly, makes full use of and shares various network resources such as existing public information networks by using virtual private network (VPN) technology. Users in different regions of the system can communicate with users in other regions of the system only by connecting with local public information network nodes, which saves investment. Virtual private network (VPN) has higher and stricter requirements for the security of network system and information. It comprehensively adopts appropriate technologies to establish separation around the internal network and external network, protect the internal network, and safely and stably protect the information platform through special firewall software, data encryption software, high-performance hardware, and comprehensive management measures.

### 2.2. Functional Module Design of Sports Physical Fitness Monitoring System

The sports physical fitness monitoring system can be divided into five functional modules: knowledge base management module, perception module, sports fitness data sampling module, fitness project information management module, and parameter setting module. These functional modules are analyzed in detail below.

#### 2.2.1. Knowledge Base Management Module

The knowledge and experience model of physical fitness analysis and evaluation experts is stored in the knowledge base, which is expressed by production rules. Production rule representation of. By analyzing the data of the inquirer, the system selects the corresponding knowledge base model and method and then generates the physical exercise methods and methods suitable for the inquirer according to the knowledge base [21, 22]. The knowledge base management system is responsible for the acquisition, retrieval, storage, and other functions of knowledge. The knowledge base also stores the technical action essentials, precautions, pictures, animations, videos of exercise methods, and diet adjustment recovered after exercise. The knowledge base is not only the organizer of sports prescription generation but also provides users with the basic knowledge and skills of physical exercise. Through learning and understanding, users can improve their interest in physical exercise, improve the quality of physical exercise, and finally achieve the effect of fitness.

#### 2.2.2. Perception Module

The core chip used in the main control board of the perception module is RK3188 with a quad-core ARM Cortex-A9 architecture of Rockchip, with the main frequency of 1.8 GHz and is equipped with the Android 4.4 operating system. Different peripherals and interface circuits are built around the system functions, as shown in Figure 2.

According to Figure 2, the main control module exchanges data with the acquisition terminal through different transmission methods such as serial port, Bluetooth, and USB and realizes the reception and transmission of human physiological parameters such as bed rest state, heart rate, pulse and respiratory rate, and measurement instructions. GPIO can realize functions such as sound acquisition output and liquid crystal display interaction. It is equipped with peripherals such as a liquid crystal display, touch screen, microphone, and speaker and uploads the monitoring data to the cloud storage platform in real time.

#### 2.2.3. Physical Fitness Data Sampling Module

The physical fitness data sampling module realizes the acquisition of video image information of the physical fitness real-time monitoring system [23], and the DM9000 network module of DAVI-COM is used to design the radio frequency interface of the physical fitness real-time monitoring system in sports training. The real-time monitoring system for physical fitness in the design of sports training is divided into four layers, which are the process management layer, AD image processing layer, parameter calculation layer, and interface information interaction layer. The circuit diagram of the physical fitness data sampling module obtained is shown in Figure 3.

#### 2.2.4. Physical Fitness Project Information Management Module

The entry of physical fitness measurement items is the preparation before sports physical fitness monitoring. The name, number, category, measurement unit, measurement instrument, measurement site, and other information of all items are recorded through the physical fitness item information management module. The system manager can view, modify, delete, and add new items at any time.

#### 2.2.5. Parameter Setting Module

The user's personal information settings are shown in Figure 4.

According to Figure 4, the setting of the user's personal information needs to determine the user's name, photo, and source, as well as the user's age and sports level. The determination of the physical fitness index monitoring index is mainly combined with the competitive ability characteristics of users to reflect the advantages and disadvantages of users' physical reserves.

### 2.3. Database Design

The database is the carrier for storing all information. The database of this system is divided into three modules: basic information database, measurement data storage database, and measurement standard comparison database.

1. *Basic Information Database*: store the basic file data of users and the basic information of testers
2. *Measurement Data Repository*: record all measurement information, including the results and scores of measurement items
3. *Measurement Standard Comparison Library*: records the normal standards of various indicators formulated by the World Health Organization, which are used to compare with the performance of the measured person, so as to obtain the performance grade and physical fitness grade of the measured person

Since more databases will cause a certain burden on the operation of the system, the reconstruction method is adopted to create a distributed database [24, 25]. The reconstruction method is to re-establish a distributed database from the overall design, including the database on each site, according to the implementation environment and user requirements of the system [26], according to the design idea and method of distributed database, and from a unified point of view, as shown in Figure 5.

The advantage of the reconfiguration method is that it can consider various problems in the distributed database according to the unified idea and effectively solve the data consistency, integrity, and reliability of the distributed database.

This completes the design of the sports fitness physique monitoring system. The system is used to monitor people's body temperature, heart rate, and other physiological parameters during sports. At the same time, the data are uploaded to the cloud service center for data monitoring and analysis to prevent people from fainting, sudden death, and other accidents during sports. The application of the system not only provides an effective means for objectively evaluating the intensity of human sports but also promotes the scientific management of people's sports, which is of great significance to promoting sports.

## 3. Real-Time Monitoring Method of Physical Fitness Based on Video Image

### 3.1. Image Acquisition of Physical Condition Monitoring

In order to realize the real-time monitoring of physical fitness, it is necessary to reconstruct the three-dimensional contour and collect the sample pixels of the sports physical fitness monitoring image in sports training [27]. The ray-casting image feature scanning method is used to collect the physical condition monitoring image in sports training. The common spatial scanning methods of physical condition monitoring image in sports training are Cell Projection and Splatting. The ZigBee video monitoring network is designed in the environment of the Internet of things [28, 29]. The physical condition video image acquisition model in sports training is shown in Figure 6.

According to the image acquisition results in Figure 6, the sparse linear equations of fitness monitoring image template matching in sports training are obtained as follows:

(1) $$\begin{array}{c} F\left(a,b\right)=h\left(a,b\right)*s\left(a,b\right)+l\left(a,b\right). \end{array}$$

Here, *h*(*a*, *b*) represents the disparity function of physical condition monitoring in sports training; the symbol *∗* represents the convolution. According to the pixel-level disparity function of sports physical fitness monitoring in sports training, information center pixel calibration and feature information adaptive weighting are performed to solve the parallax template function of physical fitness monitoring in sports training. The subpixel level matching is performed on the feature segmentation regions of the physical fitness monitoring images in sports training [30, 31], and the pixel disparity of the physical fitness monitoring image distribution in sports training is obtained as follows:

(2) $$\begin{array}{c} F\left(a,b\right)=\frac{s\left(a,b\right)+l\left(a,b\right)}{w\left(a,b\right)}. \end{array}$$

Here, *w*(*a*, *b*) represents the weight coefficient of physical condition monitoring in sports training [32]. The estimated value of edge pixels for physical condition monitoring is

(3) $$\begin{array}{c} \hat{s}\left(a,b\right)=R_{k}S\left(a,b\right)+\frac{1}{C_{i}}\phi^{2}. \end{array}$$

Here, *S*(*a*, *b*) represents the pixel value of the strong texture set of the physical fitness monitoring image in sports training about the scanning point (*a*, *b*); *R*_*k*_ represents the weak texture set of the sports physical fitness monitoring part; *ϕ*^2^ represents the local variance; *C*_*i*_ represents the classification pixel set of the physical fitness monitoring image feature information in sports training. *s*_1_(*x*) and *s*_2_(*x*) are used to denote the gray value of the reconstructed image of the physical condition monitoring image in the exercise training of young children.

The spectral feature quantity of video surveillance is initialized, a real-time monitoring model is constructed, and combined with the 3D data distribution of the 3D reconstruction of the exercise training video image, the image reconstruction processing of the physical condition monitoring in the exercise training is carried out, thereby realizing the video image acquisition of the physical condition in the exercise training.

### 3.2. Physical Condition Monitoring

Because the human body's physical fitness target frame provided by the traditional method is not accurate enough, it is not suitable for the key point calibration of the physical condition monitoring image. The research shows that the slight movement of the human body target frame will seriously affect the key point calibration result. Therefore, this paper proposes to give the image convolutional cropping, translation, scaling, and rotation characteristics through the spatial transformation network, so that the moving target has spatial invariance, and the image data can be automatically spatially transformed to generate a high-quality human target frame.

Mathematically, the spatial transformation network can be regarded as a two-dimensional affine transformation [33, 34], which can be expressed as follows:

(4) $$\begin{array}{c} \left(\begin{array}{c} a_{i}^{2}\\ b_{j}^{2} \end{array}\right)=\left[\alpha_{1},\alpha_{2},\alpha_{3}\right]\times \left(\begin{array}{c} a_{i}^{f}\\ b_{j}^{f} \end{array}\right). \end{array}$$

Here, *α*_1_, *α*_2_, and *α*_3_ represent two-dimensional vectors; (*a*_*i*_^2^, *b*_*j*_^2^) represents the coordinates before the transformation; (*a*_*i*_^*f*^, *b*_*j*_^*f*^) represents the coordinates after the transformation.

After the spatial transformation network, a human body physical fitness motion pose estimation network is formed, which is used to perform preliminary pose estimation of the human body target frame. At this time, the generated pose needs to be mapped to the original human body target frame image. Naturally, an inverse spatial transformation network is required to remap the estimated human pose back to the original image coordinates.

The spatial inverse transformation network performs inverse transformation by calculating the threshold value *ϑ*and generates a grid based on the threshold value *ϑ*. The calculation method can be expressed as follows:

(5) $$\begin{array}{c} \left(\begin{array}{c} a_{i}^{f}\\ b_{j}^{f} \end{array}\right)=\left[\vartheta_{1},\vartheta_{2},\vartheta_{3}\right]\times \left(\begin{array}{c} a_{i}^{2}\\ b_{j}^{2} \end{array}\right). \end{array}$$

Here, (*a*_*i*_^*f*^, *b*_*j*_^*f*^) and (*a*_*i*_^2^, *b*_*j*_^2^) are the coordinates before and after the spatial inverse transformation network transformation, respectively. Since the spatial inverse transformation network is the inverse process of the spatial transformation network, it can be derived as follows:

(6) $$\begin{array}{c} \left[\vartheta_{1},\vartheta_{2}\right]={\left[\alpha_{1},\alpha_{2}\right]}^{-1},\\ \vartheta_{3}=-1\times \left[\vartheta_{1},\vartheta_{2}\right]\alpha_{3}. \end{array}$$

Then, a loss function *∂*(*x*) is set, which can be deduced as follows for *α*_1_ and *α*_2_ when back propagating in the spatial inverse transformation network:

(7) $$\begin{array}{c} \partial \left(x\right)=\frac{1}{\mu \alpha_{1}}+\frac{G_{1}\left(\left(1/\alpha_{2}\right)+Y_{1}\right)}{G_{2}+\left(1/\alpha_{1}\right)+Y_{2}}. \end{array}$$

Here, *μ* represents the attitude error of the back-propagation center position of the space transformation network; *G*_1_ and *G*_2_ both represent the similarity between poses; *Y*_1_ and *Y*_2_ both represent the reference pose.

For *α*_3_, the equation can be derived as follows:

(8) $$\begin{array}{c} \partial \left(x\right)=\frac{\partial \left(x\right)}{\alpha_{3}}\times \frac{\lambda \alpha_{3}}{\lambda \vartheta_{3}}. \end{array}$$

During network training, the spatial inverse transformation network and the single-person pose estimation network are fine-tuned together.

According to the above-given derivation results, the corner detection method is used to calibrate the characteristic key points of the video surveillance part of the motion training. The expression of the corner calibration is

(9) $$\begin{array}{c} \left\{\begin{array}{c} D_{1}=\max\left({\hat{z}}_{i}-z_{i}\right),\\ D_{2}=\min\left({\hat{z}}_{i}-z_{i}\right). \end{array}\right. \end{array}$$

Here, *D*_1_ and *D*_2_ represent the image pixel difference feature quantity in the secondary matching template. The Harris corner detection method is used to locate the key feature points of the physical condition monitoring image in exercise training, and the positioning output vector is obtained as follows:

(10) $$\begin{array}{c} W_{ij}=\eta \left(a_{i}\right)\eta \left(b_{j}\right). \end{array}$$

According to the dynamic distribution of the corners of the sports physical fitness monitoring images during exercise training, the sports physical fitness monitoring is realized.

### 3.3. Recommended Fitness Methods

After the sports physical fitness monitoring is realized, the monitoring data is used as the basis, and the fitness method recommendation method is designed according to the physical fitness state of the user [35, 36], so as to improve the practical application value of the system. The following are the recommended steps for specific fitness methods:

1. Use the browser as the interaction layer, provide a data input interface and data upload function, and transmit the physical fitness test data of individual users to the WEB server;
2. The server analyzes the physical fitness test data and transmits the physical fitness test indicators after the analysis to the data mining engine. During this stage, for the acquired physical fitness test indicators, in the background database, the data mining engine matches them with the fitness categories in the fitness mode recommendation model and generates the mining results of fitness mode recommendation;
3. Send the mining results to the WEB server;
4. Individual users will be able to view the mining fitness results through their browsers.

The design of embedding the fitness mode recommendation model into the service application platform focuses on the operation phase of importing the model into the data mining engine and background database.

Import the fitness recommendation model into the database: the model and rule set are processed in a certain format and imported into the database, or the model and the database are connected using a port. The physical fitness test sample data is mined through the data mining engine, and after completion, the mining results are matched with the background fitness method recommendation table to form a recommendation list, which is presented to individual users through the browser. In this way, different users and at different times, individual users see different content on their browsers. Therefore, the fitness mode recommendation based on the individual user's physical fitness test information is realized.  Figure 7 is a flowchart of fitness mode recommendations.

## 4. Experimental Analysis

In order to verify the effectiveness of the cloud storage-oriented sports physical fitness monitoring system, an experimental study is carried out. Configure the relevant experimental parameters according to Table 1 to complete the construction of the basic experimental environment.

The storage space occupied by the compressed electric information can reflect the redundancy degree of information parameters. Generally, the smaller the storage space occupied by the compressed sports fitness monitoring system information, the lighter the redundancy degree of information parameters. At this time, the network host is more capable of eliminating redundant data.

### 4.1. Test Index Object Setting

Set the experimental test index object: take the autonomous fitness monitoring system based on a monocular camera (system 1) and the video monitoring system for children's sports training based on feature moving frame difference scanning and adaptive compensation (system 2) as the comparison system to compare with the proposed system. In the system application performance test, the focus of the test is to verify whether the accuracy and response speed of the system monitoring results meet the actual use requirements of users and the comprehensiveness of the monitoring results.

### 4.2. Analysis of Test Results

#### 4.2.1. System Response Speed

In order to verify the application effect of the monitoring system, the system response speed is used as an evaluation index. The faster the system response speed, the better the system application effect is, which indicates that the system can effectively meet the requirements of real-time monitoring of physical fitness status. Using system 1, system 2, and the proposed system to compare, the response speed comparison results of different systems are shown in Figure 8.

According to Figure 8, the response time of different systems increases with the increase of the number of experiments. When the number of experiments is 5, the response time of system 1 is 5.4 s, that of system 2 is 4.8 s, and that of the proposed system is only 2.9 s; When the number of experiments is 15, the response time of system 1 is 5.8 s, that of system 2 is 5.6 s, and that of the proposed system is only 3.3 s. Therefore, the monitoring time of the proposed system is less, indicating that the monitoring response of the proposed system is more timely.

#### 4.2.2. Accuracy of Monitoring Results

In order to verify the monitoring effect of the proposed system, the accuracy of the monitoring results is taken as the evaluation index. The higher the accuracy of the monitoring results, it shows that the system can effectively meet the actual needs of sports physical fitness monitoring, obtain accurate monitoring results, and provide reliable data for the recommendation of fitness methods. Compare system 1, system 2, and the proposed system and get the monitoring results of different systems. The accuracy comparison results are shown in Figure 9.

According to the analysis of Figure 9, with the increase of the number of experiments, the accuracy of monitoring results of different systems decreases. When the number of experiments is 5, the accuracy of monitoring results of system 1 is 60% and that of system 2 is 57%. The accuracy of the monitoring results of the proposed system is 84%; when the number of experiments is 15, the accuracy of monitoring results of system 1 is 41%, that of system 2 is 44%, and that of the proposed system is 74%. It can be seen that the accuracy of the monitoring results of the proposed method is high, and more accurate monitoring results can be obtained.

#### 4.2.3. Comprehensiveness of Monitoring Results

In order to further verify the monitoring effect of the proposed system, the comprehensiveness of the monitoring results is taken as the evaluation index. The index is expressed by numerical value, and the interval is [0, 1]. The larger the value is, the more comprehensive the monitoring results are. The monitoring results of different systems are shown in Table 2.

According to the data in Table 2, the highest comprehensive coefficient of the monitoring results of the proposed system is 9.6, and the highest comprehensive coefficient of the monitoring results of system 1 and system 2 are 7.5 and 8.0, respectively. Through comparison, it can be seen that the comprehensiveness coefficient of the proposed system is higher, indicating that its monitoring results are more comprehensive.

To sum up, with the increase of the number of experiments, the monitoring time of the sports fitness monitoring system designed for cloud storage is less, and the monitoring response is more timely; the accuracy of monitoring results is high, and more accurate monitoring results can be obtained. The highest comprehensive coefficient of the monitoring results of the proposed system is 9.6, and the comprehensive coefficient is higher, indicating that the monitoring results are more comprehensive.

## 5. Conclusion

In order to improve the accuracy of sports fitnessmonitoring results, the response speed of the system, and the comprehensiveness of monitoring results, a sports fitness monitoring system for cloud storage is designed. Based on cloud storage technology, establish the overall architecture of sports fitness monitoring system, ensure the safe and reliable transmission of fitness monitoring information under the system application support platform, and improve the accuracy of testing results; analyze the function of the hardware module of the monitoring system and establish a distributed database to improve the comprehensiveness of the detection results; ray casting image feature scanning method is used to collect the monitoring image of physical condition, and a high-quality human body target frame is generated through the steps of image convolution, cutting, translation, scaling, and rotation to realize the monitoring of the physical condition. The following conclusions are obtained through the research:

1. The physical fitness monitoring system designed for cloud storage can improve the real-time response speed of monitoring
2. Based on the monitoring data, the fitness mode recommendation method is designed according to the user's physical condition, so as to improve the application value of the system
3. The monitoring results of the designed system are more accurate, the system response speed is faster, the monitoring results are more comprehensive, and the highest value reaches 9.6, indicating that the application value of the proposed system is higher

## Figures and Tables

**Figure 1:** Schematic diagram of the overall architecture of the sports fitness monitoring system.

**Figure 2:** The working principle of the perception module.

**Figure 3:** Circuit diagram of physical fitness data sampling module.

**Figure 4:** User personal information settings.

**Figure 5:** Distributed database.

**Figure 6:** Image acquisition model of physical condition monitoring.

**Figure 7:** Fitness method recommendation process.

**Figure 8:** Response speed comparison results.

**Figure 9:** Comparison of accuracy of monitoring results.

**Table 1:** Experimental parameter setting.

Number	Equipment or indicators	Model parameter
1	Monitoring system transformer	1500 kV
2	Monitoring system substation host	IdeaCentre K350
3	Rated voltage of monitoring system	380 V
4	Rated current of monitoring system	≤51 A
5	Monitoring system resistance	6.8 × 10^7^ Ω
6	Total power consumption information storage of monitoring system	128 Gb

**Table 2:** Comprehensive comparison of monitoring results.

Number of experiments/time	The proposed system	System 1	System 2
2	9.6	7.5	8.0
4	9.4	7.3	7.9
6	9.2	7.2	7.8
8	8.9	7.6	7.5
10	9.0	7.9	7.4
12	9.0	7.1	7.5
14	8.7	7.0	7.3
16	8.7	6.8	7.1
18	9.1	7.0	7.0
20	9.3	7.0	6.9

## Data Availability

The raw data supporting the conclusions of this article will be made available by the authors, without undue reservation.
